# Anti-inflammatory and Immunomodulatory Properties of *Lepidium sativum*

**DOI:** 10.1155/2022/3645038

**Published:** 2022-07-23

**Authors:** Saeid Vazifeh, Parya Kananpour, Mahna Khalilpour, Sajjad Vazifeh Eisalou, Michael R. Hamblin

**Affiliations:** ^1^V. N. Karazin Kharkiv National University, Kharkiv, Ukraine; ^2^Laser Research Centre, Faculty of Health Science, University of Johannesburg, Doornfontein 2028, South Africa; ^3^Radiation Biology Research Center, Iran University of Medical Sciences, Tehran, Iran

## Abstract

**Background:**

*Lepidium sativum* (garden cress) is a member of the Brassicaceae family that has been utilized for medicinal and culinary purposes in centuries. Anti-inflammatory, antioxidant, immunomodulatory, hepatoprotective, antihypertensive, antiasthmatic, and hypoglycemic properties are found in various portions of the plant. The anti-inflammatory, antioxidant, and immunomodulatory effects of L. sativum were the subject of this review.

**Methods:**

The required information was gathered by searching the Web of Science, PubMed, and Scopus databases for the terms anti-inflammatory, antioxidant, immunomodulatory, immune system, and *Lepidium sativum*. Up until February 2022, the search was conducted.

**Results:**

TNF-, IL-6, IL-1, NO, iNOS, and HO-1 levels were reduced, indicating that *L. sativum* has anti-inflammatory and immunomodulatory properties. Flavonoids, alkaloids, cyanogenic glycosides, tannins, glucosinolates, sterols, and triterpenes are the key chemical components that contribute to the anti-inflammatory effects. In peritoneal neutrophils, *L. sativum* reduced oxidative stress by scavenging free radicals, as evidenced by a drop in superoxide anion and an increase in glutathione.

**Conclusion:**

The anti-inflammatory, antioxidant, and immunomodulatory activities of *L. sativum* could be explored in clinical trials to treat inflammatory and immune system illnesses.

## 1. Introduction

*Lepidium sativum* is a relatively fast-growing herb, which belongs to the family *Brassicaceae*. Garden cress is genetically related to watercress and mustard cress, sharing their peppery, tangy flavor, and aroma. In some regions, garden cress is known as “mustard and cress,” “garden pepper cress,” pepperwort, pepper grass, or poor man's pepper [1, 2]. This annual plant can reach a height of 60 cm (24 in), with many branches on the upper part. The white to pinkish flowers are only 2 mm (1/12 in) across, clustered in small branched clusters [3, 4]. This plant is distributed widely in Asia (Kuwait, Oman, Saudi Arabia, United Arab Emirates, Yemen, Afghanistan, Iran, Iraq, Palestine, Jordan, Lebanon, Syria, Turkey, Pakistan, China, Japan, India) [5]. The parts used medicinally are the leaves, flowers, seeds, and oils [6–9] (Figure 1).

The various parts of *L. sativum* are also used to treat throat diseases, asthma, headache, uterine tumors, nasal polyps, breast cancer [6], jaundice, liver problems, spleen and gastrointestinal disorders [10], and bone fracture healing [11]. The plant has been shown to possess antipyretic, analgesic, coagulant [6], antihypertensive [12], diuretic [13], antiasthmatic [14], hypoglycemic, antioxidant [15], and anti-inflammatory [6, 16] properties. In traditional medicine, *L. sativum* is used to treat inflammatory diseases, including diabetes mellitus, arthritis, and hepatitis [17, 18]. *L. sativum* leaves show antioxidant and anti-inflammatory effects due to the presence of sulforaphane, glucosinolate, and flavonol compounds [19]. *L. sativum* seeds show antioxidant and anti-inflammatory effects due to containing alkaloids, coumarin, flavonoids, tannins, triterpenes, 5,6-dimethoxy-2,3-methylenedioxy-7-C-*β*-D glucopyranosyl isoflavone, phenolic compounds, butylated hydroxytoluene, phytol, acetamide, oleic acid, octadecadienoic acid, sinapic acid, benzyl isothiocyanate, sterols, and glucosinolates [18, 20–27]. *L. sativum* seeds contain 24% oil, composed mainly of *α*-linolenic acid (32%) and linoleic acid (12%). This oil is reactively stable due to a high concentration of antioxidants and phytosterols [28, 29]. In an animal study, *L. sativum* oil was found to reduce lymphocyte proliferation and the production of inflammatory mediators by peritoneal macrophages [30]. A different study found that the feeding of Wister rats with a diet with *L. sativum* oil for 60 days increased tocopherol levels and antioxidant enzyme activity [31].

The present review focuses on the therapeutic potential of *L. sativum* and its constituents, due to their antioxidant, anti-inflammatory, and immunomodulatory properties.

## 2. Methods

The data of the current review article were collected from papers published up to February 2022 in databases including Web of Science, MEDLINE, Scopus, and PubMed. The searched keywords were “*Lepidium sativum*,” “*Lepidium sativum* seeds,” “anti-inflammatory effect,” “immunomodulatory effect,” and “antioxidant effect.”

## 3. Results

### 3.1. Constituents of *Lepidium sativum*

The chemical components of various parts of *L. sativum* are summarized in Table 1. More than eighty separate compounds have been identified in *L. sativum*. The steryl ester, stigmast-5-en-3*β*,27-diol-27-benzoate is a major constituent of *L. sativum* aerial parts. Moreover, alkaloids and flavonoids are major constituents of the plant seeds [32]. The seed oil of *L. sativum* contains mainly 7,10-hexadecadienoic acid, 11-octadecenoic acid, 7,10,13-hexadecatrienoic acid, and behenic acid [33].

The percentage of the main components in various part of *L. sativum* has been reported to be different in various studies. For example, the oleic acid content of *L. sativum* seed oil was reported to be 22% in the study by Diwakar et al. (2010), while in the study by Zia-Ul-Haq et al. (2012), it was 30.50%, and in the study by Mohammed (2013), it was 26.42% [34]. Therefore, in this review, we do not generally provide percentages.

According to the literature review, some studies indicated that the geographic origin of the plants, growing conditions, and environmental factors could all affect the profile of the chemical components of *L. sativum*. For example, the glucosinolate profiles were dependent on the genotype of the species, the environmental conditions during the growing period, the developmental stage of the plants, and the storage conditions between harvest and analysis [35–39].

Furthermore, some studies have suggested that the extraction procedure can significantly affect the chemical constituents of *L. sativum* [40, 41]. For instance, Abdulmalek et al. indicated that an ethanol extract of the seeds contained the highest percentage of phenolic and flavonoid compounds, as well as antioxidant capacity, compared to an aqueous extract [40]. Moreover, Aydemir and Becerik compared phenolic contents and antioxidant activity of different extracts of *L. sativum* seeds. They concluded that methanol extracts of *L. sativum* seeds had the highest phenolic contents and antioxidant activity compared with ethanol or water extracts [41]. On the other hand, it was reported that the antioxidant and anti-inflammatory activities of *L. sativum* were dose-dependent [33, 42].

To the best of our knowledge, there has not been any review about the anti-inflammatory, antioxidant, and immunomodulatory effects of *L. sativum*. The novelty of the present review is that it examines the anti-inflammatory, antioxidant, and immunomodulatory effects of *L. sativum* and its constituents in laboratory models, both in vitro and in vivo.

### 3.2. Antioxidant and Anti-inflammatory Effects

Highly reactive free radicals and reactive oxygen species (ROS) are normally produced in most biological systems. These ROS can lead to the oxidative damage of nucleic acids, proteins, and lipids, thus producing DNA mutations and degenerative diseases [46]. Antioxidants can trap these free radicals and quench the ROS. Antioxidant compounds like phenolic acids, polyphenols, and flavonoids can scavenge free radicals such as hydroxyl, hydroperoxide, and lipid peroxyl radicals, as well as quenching hydrogen peroxide and superoxide anion, thus inhibiting the oxidative damage that leads to degenerative diseases [47, 48].

Oxidative stress is often associated with nitrosative stress caused by production of NO and reactive nitrogen species, which are major initiators of inflammation and proinflammatory signaling [49]. Thus, antioxidants can be considered as anti-inflammatory molecules. Some studies have demonstrated the antioxidant activity of *L. sativum* seed extracts in different solvents, which can prevent inflammation [50, 51].

### 3.3. Anti-inflammatory Effects of *Lepidium sativum* Leaf Extracts

Malar et al. assayed the antioxidant activity of different parts of the plant *L. sativum*. They reported that the content of reduced glutathione in the ethanolic extracts of *L. sativum* (10 mg/mL) was higher in the leaves than in the other parts of the plant. This study showed that the scavenging activity of the leaf extract was more effective than the seeds [52]. An in vitro study by Türkoğlu et al. investigated the effects of *L. sativum* leaf extract on human keratinocyte cells. They showed that this extract (10 g/100 mL) altered the expression levels of several genes, including vascular endothelial growth factor (VEGF), tumor necrosis factor-alpha (TNF-*α*), and 5 alpha-reductase type II (SRD5A2) in cultured keratinocyte cells [53].

### 3.4. Anti-inflammatory Effects of *Lepidium sativum* Seeds

#### 3.4.1. Lepidium sativum Seed Powder

Ahmad et al. investigated whether polysaccharides contained in *L. sativum* seed powder (at doses of 250 or 500 mg/kg) had any effect on TNF-*α* production in *Escherichia coli*-stimulated mice. They showed that the polysaccharides in this plant had a significant inhibitory effect against *E. coli*-induced inflammation by reducing the circulating levels of TNF-*α* [54]. Raval et al. evaluated the effects of *L. sativum* seed powder (550 mg/kg) in Charles Foster albino rats on fibroblasts and connective tissue. Inflammation was induced by subcutaneous injection into the left hind paw of carrageenan (acute inflammation) or formaldehyde (chronic inflammation). They found that *L. sativum* has a strong inhibitory effect on the proliferation of fibroblasts and modulated the formation of connective tissue [16].

#### 3.4.2. Lepidium sativum Seed Extracts

Fan et al. isolated two new acylated flavonol glycosides from the seeds of *L. sativum*, called “kaempferol-3-O-(2-O-sinapoyl)-*β*-D-galactopyranosyl-(1 ⟶ 2)-*β*-D-glucopyranoside-7-O-*α*-L-rhamnopyranoside” and “quercetin-3-O-(6-O-benzoyl)-*β*-D-glucopyranosyl-(1 ⟶ 3)-*β*-D-galactopyranoside-7-O-*α*-L-rhamnopyranoside.” These researchers found that the two new compounds could both inhibit NO production in a macrophage cell line [55].

Tounsi et al. carried out an in vitro study which demonstrated that *L. sativum* extract (0.016 and 0.16 mg/mL) could prevent the production of superoxide anion in peritoneal neutrophils obtained from BALB/c mice, in a dose-dependent manner. It also increased glutathione and nitric oxide levels. They suggested that the flavonoids could act as an antioxidant to inhibit ROS production, scavenge and neutralize ROS and free radicals, preserve the levels of reduced GSH, and prevent oxidative damage of biomolecules [42]. Attia et al. suggested that a methanol extract of *L. sativum* seeds could control diabetes, through an antioxidant effect and improving the lipid profile. They showed that the pancreatic tissue removed from diabetic rats showed inflamed acinar tissue (lymphocytes and eosinophils between islet cells) and marked inflammation in the ducts, whereas treatment with *L. sativum* at 100 mg/kg showed improved tissue histology with few lymphocytes between islet cells. *L. sativum* treatment at 200 mg/kg showed few lymphocytes at the periphery of the islets and no inflammation around large ducts. Moreover, *L. sativum*-treatment at 300 mg/kg showed no evidence of inflammation, and the pancreatic tissues were restored to normal. They concluded that *L. sativum* methanol extract had an antidiabetic, anti-inflammatory, and antioxidant activity in a dose-dependent manner [56]. They carried out a histopathological study to assess the effect of a *L. sativum* seed ethanolic extract (150 and 300 mg/kg) in rats with liver damage induced by administration of D-galactosamine-/lipopolysaccharide. The *L. sativum* seed ethanolic extract attenuated acute necrosis and inflammation in the liver tissue [57].

A study conducted by Rajab and Hatem investigated the efficacy of *L. sativum* seeds at a dose of 200 mg/kg daily for twelve weeks against carbon tetrachloride- (CCl_4_-) induced hepatotoxicity in rats. The CCl_4_ treated rats showed a marked increase in the serum levels of liver enzymes (GOT, GPT, and ALP), a decrease in antioxidants (GSH and CAT), and severe pathological damage to liver tissue. These rats showed degenerated liver cells, thickened central vein walls, and inflammatory cells in the portal tracts and central veins. The ethanolic extract of *L. sativum* seeds could reduce the liver enzymes, increase antioxidant levels, and ameliorate the pathological damage [58]. Kadam et al. evaluated the anti-inflammatory potential of the *L. sativum* seed extract, using a human red blood cell membrane stabilization assay and a protein denaturation inhibition assay. The percent membrane stabilization for *L. sativum* seed extract was studied at various doses (50–250 *μ*g/mL). The results showed that this extract could increase 2,2-diphenyl-1-picrylhydrazyl (DPPH), 2,2′-azino-bis (3-ethyl-benzothiazoline-6-sulphonic acid (ABTS)), and superoxide anion radical scavenging activity, thereby inhibiting the production of autoantigens and denaturation of proteins. Analysis of the extract confirmed the presence of many bioactive compounds, such as coumaroylquinic acid, apigenin 6-C-glucoside, quercetin, caffeoylquinic acid, kaempferol, coumaroylquinic acid, p-coumaroyl glycolic acid, and caffeic acid [59]. Selek et al. investigated the antioxidant and anticancer effects of *L. sativum* seed methanolic extract (100, 200, and 300 *μ*g/mL) on colon and endometrial cancer cells using CUPRAC and ABTS radical scavenging activity assays. They showed that the plant extract was cytotoxic to cancer cells in a concentration-dependent manner due to its antioxidant properties [60]. Al-Sheddi et al. investigated the protective effects of a chloroform extract of *L. sativum* seeds (5–500 *μ*g/mL) against oxidative stress and cytotoxicity induced by H_2_O_2_ in human liver cells, using MTT, neutral red uptake, and morphological assays. The results demonstrated that *L. sativum* significantly improved H_2_O_2_-induced loss of cell viability up to 48%. Also, it inhibited the generation of ROS and lipid peroxidation and increased the mitochondrial membrane potential and GSH levels [61].

Hadj et al. identified the main flavonoid compounds in *L. sativum* extract present at high concentrations, such as flavonols (quercetin, kaempferol), flavones (luteolin, apigenin), and flavanones (naringin, naringenin) using high-performance liquid chromatography with diode array detection (HPLC-DAD). Biochemical and histopathological examinations revealed the protective effects of *L. sativum* flavonoid-rich extracts on high-fat diet-fed Wistar rats. They suggested that flavonoids could improve insulin sensitivity, dyslipidemia, inflammation, and pancreatic *β* cell viability [62].

Yadav et al. designed a study to investigate the potential nephroprotective activity and antioxidant potential of 200 mg/kg and 400 mg/kg ethanolic extract of *L. sativum* seeds against cisplatin-induced nephrotoxicity in albino rats. Cisplatin led to body weight loss, increased urine excretion, and increased urea and creatinine levels in serum. These changes were significantly reversed by *L. sativum* extract. Cisplatin increased malondialdehyde, superoxide dismutase, catalase, and reduced glutathione levels in kidney tissue, while these were significantly ameliorated in the *L. sativum* group. Liver enzymes, including Na^+^/K^+^ ATPase, Ca^++^ ATPase, and Mg^++^ ATPase, were significantly elevated after cisplatin injection, while these were lowered by *L. sativum* treatment. They concluded that cisplatin-induced nephrotoxicity was due to oxidative stress, and the ethanolic extract of *L. sativum* seeds could be nephroprotective [12]. Zamzami et al. showed that an aqueous extract of *L. sativum* seeds (200 and 400 mg/kg) could reverse the hepatotoxic effects of CCl_4_ and improve liver function in New Zealand white rabbits. *L. sativum* seed administration normalized the level of oxidative stress. The CCl_4_ treated group showed a suppressed antioxidant system in the liver tissue, with abnormal histopathologic changes which were reversed by *L. sativum* [20]. Sakran and colleagues reported that a methanolic extract of *L. sativum* (60, 95, or 126 mg/kg) could protect the liver against hepatotoxicity induced by paracetamol in Sprague Dawley rats [18].

Another study by Al-Asmari et al. showed that *L. sativum* seed ethanolic extract (100, 200, and 400 mg/kg) had hepatoprotective activity against CCl_4_ in Wistar rats, which was attributed to the presence of anti-inflammatory compounds and antioxidant activity. They analyzed *L. sativum* seeds using GC-MS and high-performance liquid chromatography. Their analysis revealed high concentrations of phenol derivatives, butylated hydroxytoluene, phytol, acetamide, hexadecanoic acid, and oleic acid in *L. sativum* seed extract [63]. After analyzing aqueous and alcoholic extracts of *L. sativum* seeds, Abdulmalek et al. found high concentrations of phenolic derivatives with anti-inflammatory properties. They found that eight weeks of oral intake (100 and 200 mg/kg) prevented the early metabolic alterations and weight gain induced by a high-fat diet in Sprague-Dawley rats. They explained this result by the presence of phenolic compounds in the extract [40]. Al-Yahya et al. showed that gastric mucosal lesions caused by indomethacin administration in mice could be improved by feeding an ethanolic extract of *L. sativum* seeds (100 mg/kg/day) for three months in drinking water. They proposed that the ethanolic extract of *L. sativum* seeds exerted a significant anti-inflammatory activity by inhibiting prostaglandin synthesis [6].

#### 3.4.3. Anti-inflammatory Effects of *Lepidium sativum* Seed Oil

An in vitro study conducted by Alqahtani et al. showed that the free radical (DPPH) scavenging activity and anti-inflammatory activity of *L. sativum* seed oil were concentration-dependent. The percent of inhibition DPPH of *L. sativum* seeds oil was 21%, 11%, and 7% for concentrations of 300, 200, and 100 *μ*g/mL, respectively [33].

Diwakar et al. demonstrated the modulatory effect of *α*-linolenic acid-rich *L. sativum* seed oil (2·5, 5·0, and 10%, *w*/*w*) on the lipid compositions, spleen lymphocyte proliferation, and inflammatory mediator production by peritoneal macrophages in female Wistar rats. The oil modulated inflammatory mediators, such as NO and LTB4, and may thus play a role in treating inflammatory conditions [30].

Reddy et al. showed that *L. sativum* seed oil (10% *w*/*w*) could improve dextran sulfate sodium-induced ulcerative colitis in Wistar rats. They reported that TNF-*α*, IL-1*β*, and leukotriene B4 were notably decreased in the rats treated with *L. sativum* seed oil. They concluded that *L. sativum* seed oil could alleviate oxidative stress, reduce inflammatory mediators, and decrease colon damage in ulcerative colitis rats [64]. Summary of anti-inflammatory and immunomodulatory *Lepidium sativum* effects is presented in Figure 2 and Table 2.

### 3.5. Clinical Studies with *Lepidium sativum*

Some clinical studies have examined the effects of *L. sativum* on various diseases in humans. For example, Maghrani et al. reported that an aqueous extract of *L. sativum* seeds could improve hypertension by increasing water and electrolyte secretion thereby decreasing blood pressure. They showed that daily oral administration of the aqueous *L. sativum* extract (20 mg/kg for three weeks) significantly decreased systolic blood pressure from the 7th day to the end of the treatment [65]. Paranjape and Mehta showed the clinical efficacy of *L. sativum* seed powder in treating bronchial asthma. They administered the powder at a dose of 1 g/thrice a day orally for four weeks to 30 patients of either sex aged 15-80 years who had been diagnosed with bronchial asthma. The results showed a significant improvement in clinical symptoms, respiratory function, and severity of asthmatic attacks. None of the patients exhibited any side effects from *L. sativum*. They proposed that *L. sativum* seeds could be beneficial in patients with bronchial asthma [14].

## 4. Discussion

This study is aimed at investigating the anti-inflammatory and immunomodulatory effects of *L. sativum*, in various laboratory studies. The in vivo models included rabbits, mice, and rats, and the in vitro studies used human cells, derived from the spleen, kidney, blood, and liver. In this section, we discuss the important mechanisms of the *L. sativum* and its components. Many of the compounds in *L. sativum* are known to have beneficial biological functions. In particular, flavonols, flavonoids, isoflavones, phenolic acids, lignans, and alkaloids have antioxidant and anti-inflammatory properties [66–69].

In the study by Türkoğlu et al., the anti-inflammatory effects of *L. sativum* leaf extract were attributed to the lowering of TNF-*α*, SRD5A2, and VEGF levels. These changes could be caused by the organosulphur and phenolic compounds of the plant, which are effective in free radical scavenging [53]. In agreement with this proposal, Ahmad et al. showed that *L. sativum* seeds reduced the inflammatory factors and TNF-*α* present in *E. coli*-stimulated mouse plasma [54].

Other studies have shown that the DPPH, ABTS, and superoxide anion radical scavenging activity could be caused by the phenolic and flavonoid contents, suggesting that *L. sativum* seeds have an antioxidant activity [52, 70, 71].

Flavonoids are known to regulate the expression of antioxidant enzymes, such as glutathione S-transferase (GST), NADH quinone dehydrogenase-1 (NQO-1), and heme oxygenase-1 (HO-1) by activating intracellular redox sensors such as nuclear factor like 2 (Nrf2) [72, 73]. This plant could scavenge ROS in order to reverse mitochondrial membrane dysfunction in H_2_O_2_ exposed human liver cells. Moreover, it inhibited hepatic MDA and lipid peroxidation induced by H_2_O_2_ [61]. On the other hand, the methanol extract of *L. sativum*, due to its high content of phenolic and flavonoid compounds, could decrease ROS and free radicals and improve mitochondrial and lysosomal activity. Accordingly, *L. sativum* exerted an anticancer effect on colon and endometrial cancer cells [60]. A review study by Tewari et al. suggested that a number of the chemical components of *L. sativum* such as quercetin and caffeic acid could prevent and treat cancer by modulating AP-1-associated signaling pathways [74]. Another review study proposed that natural products were a good source of novel active agents, especially when coupled with synthetic chemistry and biology, allowing the discovery of novel structures that can effectively treat a variety of human diseases [75].

It has been reported that two new flavonol compounds called “kaempferol-3-O-(2-O-sinapoyl)-*β*-D-galactopyranosyl-(1 ⟶ 2)-*β*-D-glucopyranoside-7-O-*α*-L-rhamnopyranoside” and “quercetin-3-O-(6-O-benzoyl)-*β*-D-glucopyranosyl-(1 ⟶ 3)-*β*-D-galactopyranoside-7-O-*α*-L-rhamnopyranoside” could prevent NO production in vitro [55]. *α*-Linolenic acid is the main component of *L. sativum* seeds which prevents NO production and inhibits inducible NO synthase gene expression. *α*-Linolenic acid may exert this function by blocking NF-*κ*B activity and the phosphorylation of mitogen-activated protein kinase (MAPK) in macrophages [76]. *L. sativum* ethanolic extract markedly reduced iNOS-2 expression and nitrate content. The decrease in nitrosative stress significantly downregulated the nuclear expression of NF-*κ*B and NF-*κ*B DNA binding activity and reduced cytokines (TNF-*α* and IL-6) in a dose-dependent manner [57]. Moreover, flavonoids can regulate the expression of antioxidant enzymes, such as glutathione S-transferase (GST), NADH quinone dehydrogenase-1 (NQO-1), and heme oxygenase-1 (HO-1) by activating intracellular redox sensors, such as nuclear factor like 2 (Nrf2) [72, 73]. Diets containing *L. sativum* seed oil can replace linoleic acid with *α*-linolenic acid and change the fatty acid composition to increase *α*-linolenic acid, eicosapentaenoic acid, and docosahexaenoic acid in the cell membrane lipids to modulate the immune response. The proliferation of peritoneal macrophages and spleen lymphocytes was inhibited, and the subsequent release of inflammatory mediators, such as leukotriene B4, NO, and TNF-*α*, was reduced [30]. It was reported that *L. sativum* seed oil contained high levels of *γ*-tocopherol (87.74 mg/100 g) [29], and it is known that *γ*-tocopherol can prevent inducible NO synthase in activated macrophages [77]. Diwakar and coworkers also proposed that the decrease in NO production in peritoneal macrophages might be due to the presence of *α*-linolenic acid and *γ*-tocopherol in *L. sativum* seed oil [30].

Carrageenan-induced edema in the rat paw increases inflammatory mediators such as histamine, serotonin, and bradykinin, while *L. sativum* treatment improved them. Possible mechanisms may include the inhibition of the production and release of inflammatory mediators, modulation of the interactions with their receptors, and blockade of receptor activity. Formaldehyde-induced rat paw edema increased the proliferation and migration of fibroblasts, while *L. sativum* treatment inhibited fibroblast proliferation and modulated the connective tissue [16].

It has been reported that *L. sativum* shows hepatoprotective effects. This was attributed to the presence of alkaloids, coumarin, flavonoids, tannin, and triterpenes which can all decrease free radical production and increase antioxidant activity. The *L. sativum* extract also downregulated mRNA expression of cytokines (TNF-*α* and IL-6) and stress genes (iNOS and HO-1) and upregulated IL-10. Furthermore, another study suggested that the isoflavonoid compounds extracted from *L. sativum* seeds, including 5,6-dimethoxy-2,3-methylenedioxy-7-C-*β*-D glucopyranosyl isoflavone could improve the lipid profile and the liver enzymes in serum by reducing free radicals and enhancing antioxidants. The level of MDA was lower, and antioxidant enzymes (GST, SOD, and CAT) were significantly increased in the *L. sativum* treated group [18, 20, 63]. Another study suggested that the antioxidant activity of aqueous and alcoholic extracts could be due to phenolic and flavonoid compounds in these seeds. These extracts significantly downregulated hepatic tissue inflammation and oxidative stress in high-fat diet rats by regulating AKT/mTOR signaling. The extracts lowered the concentration of AGEs (advanced glycation end products) in serum and liver tissue of *L. sativu*m seed-treated rats in an experimental study. The increase in hepatic proinflammatory markers, including TNF-*α*, IL-1*β*, IL-6, and iNOS, in high-fat diet rats was alleviated by *L. sativum* seed extract [40]. An ethanolic extract of this plant exerted significant anti-inflammatory effects by inhibiting prostaglandin synthesis in the gastric tissue of rats [6].

Aydemir and Becerik suggested that the presence of phenolic compounds in the methanol, ethanol, and aqueous extracts of *L. sativum* seeds could be an explanation of their antioxidant activity. Phenolic compounds can chelate free iron and prevent radical oxidative chain reactions in biological systems, while the scavenging activity also increases [41].

*L. sativum* leaves contain tocopherol, tocotrienols (vitamin E), phenolic compounds, nitrogen compounds, terpenoids, and other metabolites with beneficial biological activities [35, 78]. Vitamin E is present in green leafy vegetables and is considered to be a strong antioxidant [79]. Some studies have shown that vitamin E can decrease the risks of infertility, neurological disorders, inflammation, cardiovascular disease, diabetes, and some cancers in humans [80, 81]. The antioxidant activity of vitamin E leads to the induction of antioxidant enzymes such as superoxide dismutase, NADPH, quinone oxidoreductase, and glutathione peroxidase and subsequently decreases free radicals and superoxide radicals [79]. The anti-inflammatory activity of vitamin E is exerted through specific mechanisms, including the transcription factor NF-*κ*B, suppressing the expression of TNF-*α*, IL-1*β*, IL-6, IL-8, iNOS, and cyclooxygenase 2, as well as suppressing the STAT3 cell-signaling pathway and hypoxia-induced factor-1 pathway [79].

## 5. Conclusions

The present review has highlighted the anti-inflammatory, antioxidant, and immunomodulatory effects of *L. sativum* and its major phytochemical components and has suggested some possible mechanisms of action. The anti-inflammatory, antioxidant, and immunomodulatory properties of *L. sativum* are due to the presence of components such as alkaloids, coumarin, flavonoids, tannins, triterpenes, isoflavonoids, phenol derivatives, butylated hydroxytoluene, acetamide, hexadecanoic acid, oleic acid, *α*-linolenic acid, and *γ*-tocopherol. Therefore, the plant and its constituents could be used to prevent or treat inflammatory diseases or disorders associated with increased oxidative stress.

## Figures and Tables

**Figure 1:** Ethnobotanical information about *Lepidium sativum*.

**Figure 2:** Summary of anti-inflammatory and immunomodulatory *Lepidium sativum* effects.

**Table 1:** The chemical components of the various parts of *Lepidium sativum*.

Part of plant	Phytochemical compounds	Ref.
Aerial parts	Glucotropoeolin; 4-methoxyglucobrassicin; sinapine; sinapic acid; quinic acid; erucic acid; calmodulin; sinapoyglucose; caffeic acid esters; P-coumaric acid; ferulic acid; 5-4′-dihydroxy-7,8,3′,5-tetramethoxyflavone; 5-3′-dihydroxy-7,8,4′-trimethoxyflavone; 5-3′-dihydroxy-6,7,4′-trimethoxyflavone; stigmast-5-en-3*β*,27-diol-27-benzoate; cardiac glycosides; alkaloids; phenolic compounds; flavonoids; cardiotonic glycosides; coumarins; glucosinolates; saponins; sterols; tannins; volatile oils; triterpenes; linolenic acid (30.2%); uric acid (3.9%); carbohydrates, proteins; vitamins; amino acids (glutamic acid, leucine, methionine); mucilage; resins	[7, 32]
Leaves	Monoethanolamine; 1-deoxy-d-mannitol; 1-nitro-2-propanol; 2-butanamine; furfural; allyl isothiocyanate; paromomycin; 2-hydroxy-2-(5-methylfuran-2-yl)1-phenylethanone; 3,6-diazahomoadamantan-9-one hydrazone; 2,3,4-trimethoxy cinnamic acid; 2,3,4,4a,5,6,7-octahydro-1,4a-dimethyl-7-(2)-2-naphthalenol; cis-vaccenic acid; 9-octadecenamide; *γ*-tocopherol; phthalic acid decyl oct-3-yl ester; ergosta-5,22-dien-3-ol acetate; campesterol; 24-propylidene-cholest-5-en-3-ol; protein; fat; carbohydrate; minerals (calcium, phosphorous, trace elements: iron, nickel, cobalt, iodine); vitamins (vitamin A, thiamine, riboflavin, niacin, ascorbic acid); glycerin	[7, 43]
Seeds	Alkaloids; lepidine; semilepidine; glucotropaeolin; N, N′-dibenzyl urea; N, N′-dibenzylthiourea; sinapic acid; sinapin; ferulic acid; *α*-linolenic acid; linoleic acid; benzoic acid; gallic acid; dihydroxy benzoic acid; vanillic acid; chlorogenic acid; 4-hydroxycoumaric acid; salycilic acid; pyrogallol; quercetin; catechol; catechin; caffeine; flavonoids; tannins; glucosinolates; sterols; triterpenes; carotene; cellulose; calcium; sulphur; phosphorus; iron; thiamine; riboflavin; niacin; uric acid; isoleucine; cyanogenic glycosides (trace)	[6, 7, 28, 29, 34, 44, 45]
Seed oil	Palmitic acid; stearic, oleic acid; linoleic acid; arachidic acid; behenic acid; lignoceric acid; benzyl isothiocyanate; benzyl cyanide; sterols; sitosterol; 10-hexadecadienoic acid; 11-octadecenoic acid; 7,10,13-hexadecatrienoic acid	[6, 7, 33, 34]

**Table 2:** Antioxidant and anti-inflammatory effects of various parts of *Lepidium sativum* plants.

Author	Extract	Constituents	Dose	Model	Effects	Ref.
Rajab and Ali	Ethanolic	—	200 mg/kg	Carbon tetrachloride/induced hepatotoxicity in rats	Reductions in GOT, GPT, ALP, GSH, and inflammatory cells Pathologic damage in liver tissue	[58]
Ahmad et al., 2018	Powder	Polysaccharides	250 and 500 mg/kg	*Escherichia coli*-stimulated mice	Reduced TNF-*α*	[54]
Kadam et al., 2018	Ethanolic	Phenolic and flavonoid compounds: kaempferol; coumaroylquinic acid; p-coumaroyl glycolic acid; caffeic acid; coumaroylquinic acid; apigenin 6-C-glucoside; quercetin; caffeoylquinic acid	50-250 *μ*g/mL	In vitro, human red blood cells	Reduced DPPH and ABTS Increased SOD	[59]
Selek et al., 2018	Methanolic	Phenolics (gallic acid); flavonoids (quercetin)	100, 200, and 300 *μ*g/mL	In vitro, human colon cancer, endometrial cancer cell lines	Increased antioxidants, proliferation, mitochondrial, and lysosomal activity Reduced apoptosis	[60]
Al-Sheddi et al., 2016	Chloroform	Phenolics, flavonoids	5–500 *μ*g/mL	H_2_O_2_-induced cytotoxicity in human liver cells	Increased cell viability, GSH, and mitochondrial membrane potential; reduced ROS and lipid peroxidation	[61]
Raval et al., 2013	Powder	—	550 mg/kg	Carrageenan and formaldehyde-induced inflammation in Charles Foster albino rats	Reduced proliferation of fibroblasts, modulated connective tissue	[16]
L'hadj et al., 2019		Flavonols (quercetin, kaempferol); flavones (luteolin, apigenin); flavanones (naringin, naringenin)		High-fat diet Wistar rats		[62]
Yadav et al., 2010	Ethanolic	—	200 and 400 mg/kg	Cisplatin-induced nephrotoxicity in albino rats	Increased glutathione, SOD, CAT, and kidney enzymes; reduced MDA	[12]
Zamzami et al., 2019	Aqueous	Alkaloids, coumarin, flavonoids, tannin, triterpenes	200 and 400 mg/kg	Carbon tetrachloride-induced hepatotoxicity in New Zealand rabbits	Reduced free radicals, TNF-*α*, IL-6, iNOS, and HO-1; increased antioxidant activity and IL-10	[20]
Sakran et al., 2014	Methanolic	Isoflavonoids	100 and 200 mg/kg/week	Paracetamol-induced hepatotoxicity in male rats	Reduced free radicals and MDA; increased GST, SOD, and CAT	[18]
Aydemir and Becerik, 2011	Methanolic, ethanolic, aqueous	Phenolic compounds	500 *μ*g/mL	In vitro	Chelated Fe^2+^; reduced DPPH and H_2_O_2_	[41]
Al-Asmari et al., 2015	Ethanolic	Alkaloids, carbohydrates, saponins, tannins, phenolics, flavonoids, *α*-linolenic acid	100, 200, or 400 mg/kg, once daily for 7 consecutive days	Carbon tetrachloride/induced hepatotoxic in Wistar rats	Reduced free radicals; increased antioxidant activity and SOD	[63]
Abdulmalek et al., 2021	Alcoholic and aqueous	Phenolic and flavonoid compounds	200 and 400 mg/kg	High-fat diet rats	Reduced free radicals, TNF-*α*, IL-6, IL-1*β*, AGES, iNOS, proinflammatory cytokines, and chemokines; increased antioxidant activity in hepatic tissue	[40]
Al-Yahya et al., 1994	Ethanolic	Alkaloids, cardiac glycosides, flavonoids, tannins, anthraquinones, saponins, sterols, triterpenes, volatiles, cyanogenic glycosides, glucosinolates	500 mg/kg	Gastric mucosal lesions induced by indomethacin	Increased anti-inflammatory mediators; reduced prostaglandin synthesis	[6]
Tounsi et al., 2019	Methanol	Aglycones, flavonoids	0.016 and 0.16 mg/mL	In vitro peritoneal neutrophils from BALB/c mice	Reduced DPPH, nitrite, and O_2_^−^; increased SOD and GSH	[42]
Diwakar et al., 2011	*L. sativum* seed oil	*α*-Linolenic acid, eicosapentaenoic acid, docosahexaenoic acid, *γ*-tocopherol	2·5, 5·0, and 10%, *w*/*w*	Female Wistar rats	Reduced leukotriene B4, NO, iNOS, and TNF-*α*	[30]
Reddy et al., 2014	*L. sativum* seed oil	*α*-Linolenic acid, tocopherols	10% for 7 weeks	Colon ulcerative colitis in female Wistar rats	Reduced TNF-*α*, IL-1*β*, leukotriene B4, MDA, and NO; increased GSH	[64]

## Data Availability

Data will be made available on request.
